# A PDCA Model for Disinfection Supply Rooms in the Context of Artificial Intelligence to Reduce the Incidence of Adverse Events and Improve the Disinfection Compliance Rate

This article has been retracted.

**DOI:** 10.1155/2022/4255751

**Published:** 2022-03-30

**Authors:** Yunxia Wang, Shuying Zhang, Mingmei Chi, Junmei Yu

**Affiliations:** ^1^The Disinfection Supply Room of Changyi People's Hospital, Changyi, Shandong Province 261300, China; ^2^Health Examination Center of Changyi City People's Hospital, Changyi, Shandong Province,261300, China; ^3^The Second Ophthalmology Department of Changyi People's Hospital, Changyi, Shandong Province,261300, China; ^4^Disinfection and Supply Department of Zibo Central Hospital of, Zibo, Shandong Province,255000, China

## Abstract

As an important section for controlling hospital infection, the main responsibility of the sterilization supply room is to clean, disinfect, sterilize, store, and distribute all medical devices that need to be reused in the hospital, and the quality of its work is closely related to the normal work of the hospital. Disinfection and supply department is the premise and foundation of the hospital department, mainly responsible for the recovery, cleaning, disinfection, sterilization, storage, and distribution of medical devices. The cleaning and disinfection work is characterized by strong technicality and high requirements, and the work effect is directly related to the safety of patients' lives and the occurrence of hospital infections. Therefore, there is an urgent need for a scientific and efficient management mode to be applied to the work of the supply room. The traditional management mode has some drawbacks, which affects the actual work of the hospital. Disinfection and supply rooms are an important part of hospital infection control and an important department to ensure the quality of health care. An effective management mode can not only improve the efficiency but also the overall quality of work, and PDCA (plan-do-check action cycle) as an advanced management mode can effectively improve the quality of management. This study investigates the effect of PDCA cycle management based on artificial intelligence algorithms in the nursing management of sterile supply rooms, and the experimental results show that the algorithm model can effectively reduce the incidence of adverse events and improve the rate of sterilization standards, which has certain practical significance.

## 1. Introduction

Hospital management includes several aspects that require the coordination and management of people, money, materials, and time to promote medical outcomes. Hospital infection management and drug management are two important elements of hospital management. With the reform of the healthcare system and the increasingly intense healthcare market environment, hospital management is facing greater challenges and therefore needs to strengthen management interventions. In order to improve the core competitiveness of hospitals, more coping strategies are proposed to promote the improvement of medical quality and safety, and human resource management strategies play an important role in optimizing the work of hospital human resource management and promoting the further development of hospitals [1–4]. PDCA cycle management is a common quality management model used in various tasks of business management, which starts from Plan, Do, Check, and This paper discusses the effect of PDCA management in hospital management, aiming to improve hospital management treatment and guarantee patient safety. The sterilization supply room is an important place for sterilization of medical items and instruments and equipment in the hospital and is the department that provides sterile items to all departments. Its main responsibility is to recycle reusable medical devices and items in the hospital and then classify, clean and disinfect them, and store and distribute them [5–7]. The work quality of the disinfection supply room will directly affect the diagnosis and treatment work of all departments in the hospital, is the premise of ensuring aseptic operation, and plays an important role in controlling hospital infection. PDCA cycle management can effectively improve the work quality, and it will be used in the disinfection supply room to further improve disinfection through comprehensive nursing management, standardize the work flow, strengthen supervision, and continuously identify problems and solve them in the work process quality and reduce the risk of surgical instrument infection. In recent years, with the increasingly strict requirements of hospital sterilization quality, many drawbacks of the decentralized management of sterilization supply rooms in the past have been gradually exposed, which not only distract the attention of medical and nursing staff but also affect the rational optimization of hospital resources. In addition, the low qualification rate of disinfection and sterilization can easily lead to risky accidents such as medical-derived infections and in serious cases, may also lead to doctor-patient disputes. Therefore, it is important to choose scientific and effective nursing management methods for sterilization supply rooms to improve the quality of sterilization and sterilization of surgical instruments and to prevent and control medical-derived infections [8–10]. In recent years, the PDCA cycle method has been widely used to achieve quality improvement and management mainly through the cycle of planning (P), execution (D), testing (C), and processing (A). Hospital sterilization supply systems are an important part of hospital work. Due to the special nature of hospital work, surgery and treatment require a sterile environment, which places high demands on the sterilization supply system and related equipment management.

The centralized disinfection management chain for repeatedly applied instruments and materials in hospitals has a very important role, and its disinfection and sterilization quality are directly related to the overall quality of medical care and have an important correlation with the incidence of medical-derived infections [11]. It is important to carry out standardized and scientific monitoring through modern monitoring means and modern monitoring equipment. Pulsed vacuum pressure steam sterilizer is the most common and reliable sterilization treatment method for hospital medical devices. In order to effectively ensure clinical sterilization treatment, the clinic should implement physical monitoring, chemical monitoring, and biological monitoring. Among them, physical monitoring is the most basic type of monitoring means, and its sterilization parameters include sterilization temperature, sterilization pressure, and sterilization time. Sterilization temperature needs to be kept strictly within the fluctuation range to meet the minimum sterilization time requirements, and the sterilized items must meet the physical monitoring before they can be continuously applied. Biomonitoring is the only method of direct microbial sterilization, including bacterial tablets and self-contained biological indicators, and is the “gold standard” for ensuring the final sterilization results [12–15]. Chemical monitoring is an effective complement to biomonitoring, applying high-speed simulated biological performance indicators to strictly monitor all key parameters of sterilization, with easy access to monitoring results, independent of condensate and other factors, so that human-induced errors can be significantly excluded. Clinical implementation of centralized sterilization management interventions (for reused instruments, reused items, etc.) is one of the important aspects of the application of modern monitoring tools, modern monitoring equipment, etc. in the development of standardized and scientific monitoring processes. The PDCA cycle management method is a new clinical management model, which has the advantages of continuity, initiative, and timeliness, and is chosen to monitor and manage the sterile supply room, which can guarantee the effectiveness of the sterile supply room to a certain extent, effectively prevent and eliminate the problem of quality decline in the sterile supply room, and actively identify and improve the problem so as to continuously improve the quality of sterilization. Clinical studies have shown that the implementation of the PDCA cycle management method has the advantages of continuity, initiative, and the whole process, which enables the continuous improvement of the quality of physical monitoring of sterilizers in clinical hospitals, thus making the monitoring of sterilization more sound [16–19]. In addition, the PDCA cycle management intervention in sterilization rooms can further enhance the adhesion and enthusiasm of sterilization members to their work and can also effectively guarantee the consistency of sterilization work in a more comprehensive manner, thus continuously improving the level of sterilization work and reducing the incidence of medical-derived infections. The results of this study showed that the experimental group had higher qualified rates of biological monitoring sterilization effect, B-D test sterilization effect, and chemical monitoring sterilization effect, suggesting that the development of PDCA cycle management method is conducive to the improvement of sterilization quality qualification rate in sterilization supply center; the staff assessment scores of the experimental group were higher, suggesting that the development of PDCA cycle management method in clinical work has obvious advantages and is conducive to the improvement of sterilization quality in sterilization supply center. The staff assessment scores of the experimental group were higher, suggesting that the PDCA cycle management method in clinical work has obvious advantages and is conducive to improving the assessment scores of departmental staff.  Figure 1 shows the search popularity of PDCA in Google, and it can be found that it has been highly regarded by the world.

As a brand-new field that has been developing rapidly for more than a decade, deep learning has received more and more attention from researchers, and it has obvious advantages over shallow models in both feature extraction and modeling, and it is a core approach in artificial intelligence. Deep learning is good at mining increasingly abstract feature representations from raw input data, which have good generalization ability. It overcomes some of the problems that have been considered intractable in AI in the past. And with the significant growth in the number of training data sets and the dramatic increase in chip processing power, it has been effective in areas such as target detection and computer vision, natural language processing, speech recognition, and semantic analysis and therefore has contributed to the development of artificial intelligence. Deep learning is a hierarchical machine learning method that includes multilevel nonlinear transformations, and deep neural networks are the main form at present. The connection pattern between neurons is inspired by the organization of the animal visual cortex, and convolutional neural networks are one of the classical and widely used structures. The local connectivity, weight sharing, and pooling operations of convolutional neural networks enable them to effectively reduce the complexity of the network, reduce the number of training parameters, make the model invariant to translation, distortion and scaling to a certain degree, and have strong robustness and fault tolerance, and are also easy to train and optimize. Based on these superior properties, it outperforms standard fully connected neural networks in a variety of signal and information processing tasks. The paper first outlines the development history of convolutional neural networks and then describes the structure of neuron model and multilayer perceptron, respectively. Then, the structure of convolutional neural networks, including convolutional, pooling, and fully connected layers, which play different roles, is analyzed in detail. Then, improved convolutional neural networks such as the net-in-network model and spatial transformation network are discussed. Also, supervised learning and unsupervised learning training methods for convolutional neural networks and some common open-source tools are introduced, respectively. In addition, the paper summarizes the applications of convolutional neural networks with the examples of image classification, face recognition, audio retrieval, ECG classification, and target detection. The integration of convolutional neural networks with recurrent neural networks is one way [20]. In order to give the reader as much reference as possible, the paper also designs and experiments convolutional neural networks with different parameters and different depths to analyze the interrelationships among the parameters and the effects of different parameter settings on the results. Finally, several problems to be solved in convolutional neural networks and their applications are given.

Today, the emergence of PDCA cycle management technology has brought more convenient and efficient services to the sterile supply room. In order to solve the current problems of difficult feature parameter extraction and traditional methods affected by interference in disinfection supply rooms, and to improve the shortcomings of existing methods in a targeted manner, this paper verifies the performance of the model by constructing a deep learning-based algorithm and by adjusting relevant network parameters and finally verifies the effectiveness of the proposed method by using it in real disinfection supply room data.

The key contribution of this research is as follows:

- Firstly, effectiveness and order of nursing management ensured by the quality management team in the planning stage.
- In the implementation stage, the quality is improved by dividing the responsibility on the one hand and other hand improving the business quality by training the staff and sterile supply room management.
- Next stage is inspection where the quality is improved by inspection and grading the nursing staff by the group of supervisory.
- Last stage is treatment stage where drawbacks of nursing stage management are identified timely and corrected through continuous work summary that increases the quality.

The rest of the paper is organized as Section 2 represents the history. The methodology is discussed in Section 3.  Section 4 talked about the experimentation and evaluation of results of this research. Finally, concluded the study in Section 5.

## 2. Related Work

### 2.1. Sterile Supply Room Management Based on PDCA Model

With the improvement of people's living standards, the strengthening of sterile supply rooms has become a major task in health care services. Effective and scientific sterile supply room management has become a major research issue for clinical staff to improve medical satisfaction, efficiency, and quality of care. The PDCA cycle [21], also known as the quality loop, was first proposed in 1950 and is a management method that allows management to become more scientific, standardized, and procedural. Planning, inspection, implementation, and processing are the four main stages of the PDCA cycle, and the PDCA cycle process is the process of repeating the above four stages, eight steps, and four stages are what the PDCA cycle goes through every time: planning—the current situation is analyzed, the problems are identified, the influencing factors and causes of the problems are analyzed, the main elements are identified, countermeasures are proposed, and the plan is formulated; implementation—the plan is analyzed, the problems are identified, and the main elements are identified. The plan is formulated; implementation—implementation of the plan; inspection—analysis and comparison of expected goals and actual results; processing—consolidation of results, standardization of experience and analysis of evaluation, and transfer of newly discovered or unresolved problems to the next cycle. The PDCA cycle, as a quality management method, is now widely used in all aspects of nursing management. The application of PDCA cycle in sterile supply room management is not only an important function but also the core content. The quality of the sterile supply room is not only related to the level of sterile supply room management and nursing quality management methods but also related to the technical level and business quality of sterile supply room personnel [22]. The implementation of the PDCA cycle in the quality management of the sterile supply room can help make the quality of the sterile supply room more scientific and effective [23]. One study reported that the PDCA cycle in the disinfection supply rooms of cardiovascular medicine and orthopedic surgery, neurosurgery, and neurology wards, where there are more critical patients, increased the satisfaction rate of disinfection supply room management and the total nursing pass rate from 67.4% to 70.0% to 96.7% and 98.7%, with statistically significant differences, indicating that the application of the PDCA cycle in the quality management of the sterile supply room was reviewed and the conclusions were consistent with the above analysis. In order to improve patient satisfaction and quality of nursing care, the eight steps and four stages of the PDCA cycle are fully utilized in the development of nursing care management programs by medical and nursing staff, and the quality of nursing care and patient satisfaction are effectively improved through four cycles in a year, which not only positively promotes quality nursing care but also optimizes the behavior and philosophy of nursing staff.  Figure 2 illustrates the sterile supply room management system.

The use of PDCA cycle management in the sterile supply room can strengthen the process of sterilization occupational hazard protection, which indicates that the scientific validity of PDCA cycle has been confirmed, and the use of PDCA cycle management can effectively improve the protection of occupational hazards of medical and nursing staff in the sterile supply room, not only to ensure the professional safety of staff but also to reduce the occurrence of occupational hazards. In the clinical teaching of various specialties, such as respiratory medicine and operating rooms, ICU, and obstetrics and emergency medicine, the scientific validity of PDCA cycle management of the disinfection supply room has been verified, and each specialty has developed the most appropriate PDCA cycle disinfection supply room teaching model by combining its own teaching reality and characteristics [24–26]. At the same time, the enthusiasm of teachers and students can be mobilized so that the comprehensive quality and professional skills of nursing students can be improved, which can effectively improve the overall level of teachers. In conclusion, PDCA is a cycle of planning, execution, checking, and action, which has the characteristics of continuity, unity, and completeness. Compared with other nursing models, PDCA is more standardized and effective. As the PDCA cycle is applicable to the management of each sterile supply room, this will not only improve the hospital sterilization quality management and safety management but also improve the teaching management of the sterile supply room, make the patient satisfaction and the work quality of medical and nursing staff improve, reduce the occurrence of medical disputes and nursing defects, and ensure patient safety, which is worthy of application and promotion.

### 2.2. Deep Learning

Achieving artificial intelligence (AI) is a long-standing common goal of mankind. With the rapid development of modern computer technology, human beings have made great progress in the field of AI. AlphaGo1, an AI robot developed by Google, has won a 3–0 victory against the world Go champion. However, in other fields, AI is still far from realizing the real sense of “machine” instead of “brain” [27]. As an important branch of AI, neural networks can replace the human brain to effectively deal with some complex problems, thus promoting the development of AI. Artificial neural networks (ANN), also known as a collection of connected units of artificial neurons, is a framework for many different machine learning-based algorithms. ANNs are inspired by the biological neural networks that form animal brains and mimic the neurons in biological brains. Each connection, like a synapse in the biological brain, can pass signals between neurons. ANNs were originally proposed so that they could solve problems in the same way as the human brain. However, over time, the focus of ANN research shifted from biology to how to make ANNs perform specific tasks. With the flourishing of modern science, technology, and hardware devices, ANNs have an increasingly important role in handling problems with large and complex data volumes. Artificial neural networks are an analog and approximation of biological neural networks, which are adaptive nonlinear dynamic network systems composed of a large number of neurons connected to each other by interconnection. The first mathematical model of neurons, the MP model, was groundbreaking and provided the basis for later research work. The learning function was added on top of the MP model, and the single-layer perceptron model was proposed, putting the study of neural networks into practice for the first time. However, the single-layer perceptron network model is not capable of handling linearly indistinguishable problems. A multilayer feedforward network-backpropagation network trained according to the error backpropagation algorithm solved some problems that the original single-layer perceptron could not solve.  Figure 3 illustrates the basic structure of RNN.

Various shallow machine learning models have been proposed one after another, the more classical ones such as support vector machines, and the traditional BP networks encounter problems of local optimum, overfitting, and gradient diffusion when increasing the number of layers of neural networks, which put the research of deep models on hold. Artificial neural networks with multiple hidden layers have excellent feature learning ability; they can effectively overcome the training difficulties of deep neural networks by “layer-by-layer pretraining,”which has led to the research of deep learning and another boom of artificial neural networks. In the layer-by-layer pretraining algorithm of deep learning, unsupervised learning is first applied to pretrain each layer of the network, and only one layer is trained unsupervised at a time, and the training result of this layer is used as the input of the next layer and then the pretrained network is fine-tuned by supervised learning (BP algorithm). This deep learning pretraining method can significantly improve the recognition or detection results in handwritten digit recognition or pedestrian detection, especially when the number of labeled samples is limited. The network structure and learning methods are included in deep learning. Currently, the commonly used deep learning models include deep confidence networks, cascaded automatic denoising coders, convolutional neural networks, etc. RNNs are a special class of neural networks in the field of deep learning with self-connections inside, which can learn complex vector-to-vector mappings. The first research on RNN was proposed by Hopfield with the Hopfield network model, which has strong computational power and associative memory function. Jordan and Elman proposed the recurrent neural network framework, called simple recurrent network, in 1986 and 1990, respectively, which is considered to be the basic version of the now widely popular RNN, and the more complex structures that have emerged since then can be considered as its variants or extensions. It has been widely used in various tasks related to time series. The network structure of an RNN is shown, which enables the network state of the previous moment to be passed to the current moment and the state of the current moment to be passed to the next moment through loop connections on the hidden layer.

The forward propagation of RNN can be expressed as follows:

(1) $$\begin{array}{c} \left\{\begin{array}{c} h_{t}=\sigma \left(W_{xh}x_{t}+W_{hh}h_{t-1}+b_{h}\right),\\ o_{t+1}=W_{hy}h_{t}+b_{y},\\ y_{t}=\text{softmax}\left(o_{t}\right), \end{array}\right. \end{array}$$

where *W*_*hh*_ is the connection weight matrix between the hidden units, *W*_*hy*_ is the connection weight matrix from the hidden unit to the output unit, and b_y_ and *b*_*h*_ are the bias vectors. The parameters required in the computation are shared, so theoretically, RNN can handle sequence data of arbitrary length. *h*_*t*_ requires *h*_*t-1*_ for the computation of *h*_*t-1*_, *h*_*t-2*_ for the computation of *h*_*t-1*_, and so on, so the state at a certain moment in RNN is dependent on all the past states. RNN can map sequence data to sequence data output, but the length of the output sequence does not necessarily coincide with the length of the input sequence, and there can be a variety of correspondences depending on the requirements of different tasks. For neural networks with recurrent structures, since the computation of the current time step depends on the output of the previous time step, for example, in LSTM units, the update of the moment gating unit depends on the hidden state *h*_*t-1*_ at time *t* - 1, which hinders the parallel processing of the sequence, where each element of the sequence must be computed sequentially. How to speed up the training of networks with recurrent structures is also a very popular research topic recently. The proposed acceleration algorithm class recurrent neural network is a sequence modeling method that uses alternating convolutional layers. It is validated in 3 tasks related to sequence data, namely sentiment classification, language modeling, and machine translation, and it obtains good acceleration while maintaining good performance. To improve the training speed of the model, the simple loop unit is proposed. In the current field of deep learning, deeper deep networks are often used in some tasks in order to improve the performance of models; however, this often also requires more computational resources and consumes more training time. SRU is a variant structure to improve the training speed of LSTM by discarding the dependencies in the loop structure. SRU simplifies the computation of the gating unit while still maintaining a strong performance capability. In the last, we have compared the literature as shown in Table 1.

## 3. Method

### 3.1. Model Architecture

The general architecture of the proposed method is shown in Figure 4 below, which is based on RNN neural networks with the addition of PDCA cycle-related elements.

### 3.2. Method Details

One of the main problems of using gradient descent methods to optimize RNNs is that the gradient may disappear rapidly as it is backpropagated along the sequence. A large amount of research work has been done to solve the training problem in RNNs, and variants of RNNs have been proposed, two of the most representative networks being the echo state network and the LSTM. The following section will focus on the network structure of the LSTM model and its properties. At present, the most widely used recurrent structure network architecture in practical applications comes LSTM model (without forgetting gate), which can effectively overcome the gradient disappearance problem existing in RNN, especially in the task of long-distance dependence performs much better than RNN, the gradient backpropagation process will not be troubled by the gradient disappearance problem again, and can accurately model the data with short-term or long-term dependence. LSTM works in basically the same way as RNN, with the difference that LSTM implements a more refined internal processing unit to achieve efficient storage and updating of contextual information. Due to its excellent nature, LSTM has been used in a large number of tasks related to sequence learning, such as speech recognition, language modeling, lexical annotation, and machine translation. LSTM is used to learn a semantic sentence vector and then the feature vector is used for document retrieval tasks in a network whose hidden layer provides a semantic representation of the entire sentence and is able to detect keywords in the sentence. A BLSTM-based language model is introduced and a word-character gate is proposed to solve the representation of unregistered words, which can be adaptively blended with word and character-level word vectors to obtain the final word vector representation. A dynamic extended tree-based BLSTM model is used for event extraction, using dynamic extended tree, lexical, and distance information for input enrichment. A memory unit and gated memory unit are introduced to preserve historical information, long-term states, and use gating to control the flow of information. In this paper, the hidden units in LSTM networks are called LSTM units, and the recurrent neural networks in which the hidden units are LSTM units are called LSTM networks or LSTM. There are three types of gating in LSTM units, which are input gates, forgetting gates, and output gates. The gating can be considered as a fully connected layer, and it is the gating that enables the LSTM to store and update information. More specifically, gating is implemented by sigmoid functions and dot product operations, and gating does not provide additional information. The general form of gating can be expressed as

(2) $$\begin{array}{c} g\left(x\right)=\sigma \left(\mathrm{Wx}+b\right), \end{array}$$

where *σ*(*x*) *=* *1*/(1+exp(−*x*)), called the Sigmoid function, is a nonlinear activation function commonly used in machine learning to map a real value to the interval 0 to 1, which is used to describe how much information passes. When the output value of the gate is 0, it means that no information passes, and when the value is 1, it means that all information can pass. The input, forgetting, and output gates are denoted by *i*, f, and *o*, respectively, ⊙ represents the corresponding elements multiplied together, and W and *b* denote the weight matrix and bias vector of the network.

The forward computation process of the LSTM in Figure 5 can be expressed as equations (3) to (5). At time step *t*, the input and output vectors of the hidden layer of the LSTM are *x*_*t*_ and *h*_*t*_, respectively, and the memory cell is ct. The input gate is used to control how much of the current input data *x*_*t*_ of the network flows into the memory cell, i.e., how much can be saved to *c*_*t*_, with the values:

(3) $$\begin{array}{c} i_{t}=\sigma \left(W_{xi}x_{t}+W_{hi}h_{t-1}+b_{i}\right). \end{array}$$

The forgetting gate is a key component of the LSTM unit that controls which information to keep and which to forget and somehow avoids the gradient disappearance and explosion problems that arise when gradients propagate backwards in time. The forgetting gate controls the self-linking unit that can decide which parts of the historical information will be discarded. That is, the information in memory unit ct-1 at the previous moment has an impact on the current memory unit *c*_*t*_.

(4) $$\begin{array}{c} f_{t}=\sigma \left(W_{xf}x_{t}+W_{hf}h_{t-1}+b_{f}\right),\\ c_{t}=f_{t}⊙c_{t-1}+i_{t}⊙\text{tanh}\left(W_{xc}x_{t}+W_{hc}h_{t-1}+b_{c}\right). \end{array}$$

The output gate controls the effect of the memory cell *c*_*t*_ on the current output value *h*_*t*_, i.e., which part of the memory cell will be output at time step *t*. The value of the output gate is shown in (4), and the output *h*_*t*_ of the LSTM unit at time step *t* can be obtained by (5).

(5) $$\begin{array}{c} o_{t}=\sigma \left(W_{xo}x_{t}+W_{ho}h_{t-1}+b_{o}\right),\\ h_{t}=o_{t}⊙\text{tanh}\left(c_{t}\right). \end{array}$$

## 4. Experimentation and Evaluation

### 4.1. Dataset

Eight disinfection supply room nurses from this department of our hospital from January to December 2018 were selected as the control group to manage the disinfection supply room with conventional nursing management methods; nine disinfection supply room nurses from this department of our hospital from January to December 2019 were selected as the observation group. There was 1 male case and 8 female cases in the observation group; age ranged from 45 to 55 years old, with an average age of (48.12 ± 4.67) years. In the control group, there was 1 male case and 7 female cases; ages ranged from 43 to 53 years, with a mean age of (48.44 ± 4.21) years. When comparing the general data of the two groups, the differences were not statistically significant (*P* > 0.05) and were comparable.

### 4.2. Comparison Method

#### 4.2.1. Control Group

The sterile supply room was managed using conventional nursing management methods. Daily work and management were carried out according to the daily workflow. The supply room staff were strictly required to study and implement the relevant regulations and workflow of the department and work according to the basic operational requirements. Strictly divide the operation area and clearly distinguish between contaminated area, clean area, and sterile storage area to avoid mixing contaminated items with sterile items. When issuing cleaning and disinfection items, the basic information of the items should be carefully checked, including name, quantity, disinfection date, shelf life, cleanliness of packaging containers, and integrity of the items, etc., and issued in place after confirmation. After the work is finished, the floor needs to be thoroughly cleaned, the table and workbench should be scrubbed with disinfectant, the workplace environment should be kept neat and hygienic, and the items should be placed in an orderly manner. Observation group: adopt the PDCA cycle method based on the intelligent algorithm proposed in this paper to manage the sterile supply room. Develop a nursing management plan (P). Improve and perfect the weak links and problems in the nursing management of the sterile supply room, develop a scientific and reasonable nursing management plan for the sterile supply room, and improve occupational protection. Fully implement the management plan into all aspects of work. In order to improve the level of disinfection technology for medical devices, items, and equipment, these instruments should be thoroughly cleaned and disinfected to ensure packaging quality and to make the equipment meet the requirements for reuse. Management plan implementation (D). In the nursing management and sterile supply room, strengthen occupational disease hazard protection and prepare protective equipment from chemical substances. Strengthen hand hygiene management and develop emergency disposal methods and measures for accidental injuries. Standardize disinfection and sterilization of medical equipment, instruments and items, and optimize the recycling process to make the process simpler, less time-consuming, and with shorter operational steps. Special contaminated entrances and passages are designed and supervised by professionals. Strictly count, classify and verify medical equipment, check and evaluate the sterilization and cleaning effect after sterilization and cleaning, and resterilize and clean those that are not qualified. Strengthen biochemical monitoring to ensure that qualified ones are sent to the sterile room for proper classification, positioning, and clear identification. Spot check the sterilization and quality of instruments. To improve the quality of sterilization, not only should we strengthen bacteriological testing but also increase the key protection areas. Strict supervision and inspection (C). Strengthen the quality and evaluation of nursing management in the sterile supply room, and understand and evaluate the current status and level of nursing management in the sterile supply room in many aspects. Conduct all-round and multiangle inspections of complication occurrences and make detailed records to facilitate future preparation for inspection. Summarize daily, weekly, monthly, quarterly, and annual work; conduct regular spot checks, inspections, and improvements; summarize and record the effects of rectification; and properly realize circular management to achieve the purpose of improving the quality of nursing management in the sterile supply room. Continuous improvement and treatment (A). Strict supervision and inspection of the management and nursing work in the sterile supply room, summarize the effect of implementing the program, learn the lessons of deficiencies as the next experience for improvement and treatment, continuously improve and enhance the quality and application value of the nursing management program in the sterile supply room, and improve the quality and level of clinical nursing management.

### 4.3. Evaluation Metrics

To compare nurses' satisfaction with the nursing management model and nurses' work standardization rate, satisfaction = (very satisfied + satisfied)/total number of cases × 100%; standardization rate = (standardized + partially standardized)/total number of cases × 100%. SPSS 23.0 statistical software was used for data analysis, and the measurement data were expressed as *x* ± *s* with the *t*-test; the count data were expressed as rate (%) with the *χ*2 test. *P* < 0.05 considered as the difference was statistically significant.

### 4.4. Results

Nurses' satisfaction with the nursing management model was higher in the observation group than in the control group, and the difference was statistically significant (*P* < 0.05) when compared between the groups, as shown in Table 2.

When comparing the work standardization rate of nurses in the sterile supply room between the two groups, the work standardization rate of nurses in the observation group was higher than that in the control group, and the difference was statistically significant (*P* < 0.05) when comparing between the groups, see Table 3.

The quality of disinfection work was significantly better in the study group than in the control group (*P* < 0.05), as shown in Table 4.

The overall management quality scores and nursing satisfaction scores of the study group were significantly higher than those of the control group (*P* < 0.05), as shown in Table 5.

## 5. Conclusion

Hospitals should pay great attention to the quality of work in sterile supply rooms to ensure medical safety. The PDCA cycle is a scientific management model that develops scientific management plans through feedback from medical staff, strictly sterilizes medical devices and related items to ensure that they are qualified before use, strengthens management during the implementation of the plan, dynamically tracks and continuously improves the plan, and effectively improves the incentive management of sterile supply rooms The application of PDCA cycle in sterile supply room nursing management is divided into four main management stages. First, in the planning stage, the order and effectiveness of nursing management is fundamentally ensured by formulating and improving the management system and establishing a quality supervision team. Secondly, in the implementation stage, on the one hand, the division of staff responsibilities can both ensure the effectiveness of quality management and promote the clarity of quality management responsibilities, which is conducive to strengthening the sense of responsibility of staff and promoting further improvement of management quality; on the other hand, by strengthening the training of staff and improving their business quality, the management quality of the sterile supply room can be further improved. Again, in the inspection stage, the overall quality inspection and grading through the supervisory group helps to improve the quality of nursing management and the quality standard and responsibility of the staff in the sterile supply room. Finally, in the treatment stage, the shortcomings in nursing management were timely identified and corrected through regular work summaries to continuously improve the efficiency and quality of nursing management in the sterile supply room. This study showed that the satisfaction and work standardization rates of nurses in the sterile supply room managed by the PDCA cycle method were higher than those of conventional nursing management, and the differences were statistically significant when compared between groups (*P* < 0.05). In conclusion, compared with the conventional nursing management model, the artificial intelligence-based PDCA cycle method proposed in this paper is significantly applied to nursing management in the sterile supply room, reducing the incidence of adverse events and improving the rate of sterilization compliance, which can significantly improve the satisfaction rate, work standardization rate, and work quality of nurses in the sterile supply room and is worth promoting.

## Figures and Tables

**Figure 1:** PDCA hot trend in Google.

**Figure 2:** Sterile supply room management system.

**Figure 3:** RNN structure details.

**Figure 4:** Model structure.

**Figure 5:** RNN model schematic.

**Table 1:** Comparison of literature in respect of results.

Author and reference	Technique	Results	Future directions
Bianchi et.al. [19]	RNN with time series prediction and problem of short-term load forecasting	Satisfactory results obtained with minimal fine-tuning of hyper parameters, but LSTM and GRU are not better than ERNN due to simple training and simple structure	Problem with gradient-based networks training is slower as the future direction for researchers

Liu et.al. [22]	RNNs with multiple equilibria	Factors affecting multiple equilibria, activation functions, and multistability and complete stability analysis for RNN	Seven directions are formulated for future investigations

Zhang et.al. [24]	RNN with time-varying delays	Estimating the L-K functional on GAS criteria of RNN delays	Less conservative criteria of GAS on RNN delays challenging till now

Our method	RNN with PDCA cycle	Good results by improving the rate of sterilization compliance, improved satisfaction rate, work quality, and work standardization	Hospital management facing greater challenges till now

**Table 2:** Comparison of nurses' satisfaction with care management models [n (%)s].

Group	*N*	Very satisfied	Satisfied	Dissatisfied	Satisfied
Control group	8	2 (25.00)	2 (25.00)	4 (50.00)	4 (50.00)
Observation group	9	5 (55.56)	4 (44.44)	0 (0)	9 (100.00)

**Table 3:** Comparison of the work standardization rate of nurses in the sterile supply room between the two groups [n (%)].

Group	*N*	Specification	Partial specification	Not standardized	Normative rate
Control group	8	2 (25.00)	3 (37.5)	3 (37.50)	5 (62.50)
Observation group	9	4 (44.44)	5 (55.56)	0 (0)	9 (100.00)

**Table 4:** Example of work quality comparison between the 2 groups (%).

Item	Control group	Study group	*X* ^2^	*P*
Qualified rate of sterilization solution concentration (*n* = 150)	134(89.33)	149(99.33)	14.030	<0.001
Qualification rate of sterilized medical items (*n* = 50)	43(90.00)	49(98.00)	4.891	0.021
Qualified rate of surgical instrument cleaning and disinfection (*n* = 100)	90(90.00)	98(98.00)	4.714	0.029
Qualified rate of hand hygiene (*n* = 150)	134(89.33)	148(98.67)	11.584	0.001

**Table 5:** Comparison of overall management quality scores and nursing satisfaction scores between the 2 groups.

Group	Number of cases	Overall management quality score	Nursing service satisfaction score
Study group	150	92.43 ± 4.21	96.75 ± 3.22
Control group	150	80.66 ± 3.02	83.92 ± 2.77
*t*		27.822	36.995
*P*		<0.001	<0.001

## Data Availability

The datasets used during the current study are available from the corresponding author on reasonable request.
